# Aging-related tumor associated fibroblasts changes could worsen the prognosis of GBM patients

**DOI:** 10.1186/s12935-020-01571-7

**Published:** 2020-10-08

**Authors:** Hongwang Song, Xiaojun Fu, Chenxing Wu, Shouwei Li

**Affiliations:** 1 Department of Emergency Medicine, Shengjing Hospital of China Medical University, Shenyang, China; 2 Department of Neurosurgery, Sanbo Brain Hospital, Capital Medical University, Xiangshanyikesong 50#, HaiDian District, Beijing, 100093 China

**Keywords:** Glioblastoma, Tumor heterogeneity, Tumor microenvironment, Tumor associated fibroblasts, Epithelial mesenchymal transition

## Abstract

**Background:**

Glioblastoma multiforme (GBM) is the most malignant tumor in human brain, with highly heterogeneity among different patients. Age could function as an incidence and prognosis risk factor for many tumors.

**Method:**

A series of bioinformatic experiments were conducted to evaluate the differences of incidence, differential expressed genes, enriched pathways with the data from Surveillance, Epidemiology, and End Results (SEER) program, the cancer genome atlas (TCGA) and Chinese glioma genome atlas (CGGA) project.

**Results:**

We discovered in our present study that distinct difference of incidence and prognosis of different aged GBM patients. By a series of bioinformatic method, we found that the tumor associated fibroblasts (TAFs) was the most crucial tumor microenvironment (TME) component that led to this phenomenon. Epithelial-mesenchymal transition (EMT) could be the mechanism by which TAFs regulate the progression of GBM.

**Conclusion:**

We have proposed a close correlation between age and GBM incidence and prognosis, and propose the underlying mechanism behind this correlation by mining different databases, which laid the foundation for future research.

## Backgrounds

Glioblastoma multiforme (GBM) is the most malignant and frequently occurring type of primary tumor in central nervous system, which accounts for more than 60% of all brain tumors in adults [1, 2]. The current treatment of GBM relies on surgical resection of gross tumor followed by radio-chemotherapy, as well as adjuvant therapy with temozolomide. Despite such variety of therapies against it, GBM is still a deadly disease with extremely poor prognosis [1, 3]. GBM patients have a median survival of approximately 14 to 15 months after the diagnosis [4]. However, although the overall prognosis of GBM patients is very poor, there is still a significant prognostic diversity among these patients. This diversity is largely due to the heterogeneity of GBM.

Tumor heterogeneity, characterized by distinct cellular or genetic alterations that occur in individual tumors originating in the same sources, as well as non-neoplasm cells involved in the initiating and progression of tumors, is one of the most important hallmarks of GBM [5, 6]. Tumor heterogeneity includes intratumoral heterogeneity [7, 8] and intercellular heterogeneity [9]. The heterogeneity in cellular level, named as inter-tumoral heterogeneity, referred to the differences among tumor cell together with an array of supportive, immunity and stromal cells, which provide a comfort environment for tumor cells to develop and grow, and further adds to the diversity of intratumoral heterogeneity [10] Intratumoral heterogeneity allows the classification of these tumors into different molecular subtypes, namely proneural (PN), classical (CL) and mesenchymal (MES) subtypes, among which MES had the poorest outcome [7]. Intercellular heterogeneity, on the other side, contains a series of non-neoplastic cells, including infiltrating and resident immune cells, stromal cells, other glial cells, extracellular matrices (ECM) and other components related to the tumor microenvironment (TME) [11]. This tumor immunology and tumor microenvironment has added another level of complexity to this phenomenon. Spotlights have been placed on various non-neoplastic constituents of the immune system, especially tumor-associated fibroblasts (TAFs) in GBM [9]. TAFs function as crucial factor constructing a microenvironment that favors tumor initiation, angiogenesis and aggressiveness of tumors through the production of multiple ECM proteins and regulatory molecules [12]. And improved understanding of TAFs biology, as well as the potential link of TAFs to other factors would offer deeper insight into how TAFs might contribute to the dynamic complexity and functional malleability of the TME in GBM.

Age had been shown to lead to the incidence, aggressiveness of tumor, and the poorer prognosis of tumor patients [13]. The connection between cancer and age has been well-documented in numerous epidemiological studies. For example, some cancers have early-life incidence peaks, such as osteosarcoma [14] and acute lymphoblastic leukemia [15]; and the incidence of testicular cancer peaks at approximately age 30 years and then sharply declines [16]. Prostate cancer patients over the age of 55 are more likely to develop tumors with characteristics associated with favorable treatment and/or survival outcomes [17]. There are many shared mechanisms between aging and tumor, such as DNA damage responses, endocrine changes, vascular ageing and angiogenesis, and the impact of aging on immune system [13]. It is well established that the immune system becomes compromised during the process of aging (known as immunosenescence), with inflammation increasing with age [18]. By contrast, immunosurveillance also becomes compromised with age [19], and this may contribute to the increased cancer development in old age. It is therefore tempting to speculate that the increased immune and other components in TME of aging tissues may favor cancer development. It had been reported that age could promotes changes in the phenotype of the TAFs, such as mitochondrial dysfunction, hydrogen peroxide production, and aerobic glycolysis, which may lead to increased DNA damage and random mutagenesis [12]. Therefore, these processes can accelerate age-related cellular damage and promotes a permissive metabolic microenvironment for cancer development and progression, which caught great attention on the link between age and TAFs during the process of tumor progression [20]. Moreover, alternation of the components in TME (TNF-α, TGF-β, etc.) of GBM may result in change of subtype and lead to differences of outcomes [10]. But until now, there is neither any direct evidence of the effect and mechanism of aging on the prognosis of GBM, nor biological mechanism behind this link between age and TAFs in GBM.

With the development of the cancer genome atlas (TCGA), Chinese glioma genome atlas (CGGA) project, as well as the establishment of Surveillance, Epidemiology, and End Results (SEER) program, we are now able to evaluate the potential impact of aging on the GBM patients’ incidence and prognosis, and to screen out the molecular mechanisms behind this impact. Herein, in our research, we provide evidences that aging could negatively influence the outcome of GBM patients. To our astonishment, the age of 40 seems to be a significant watershed of the prognosis. We then discovered that TAFs were the only components that were significantly different between over and under 40 years old patients. By multiple bioinformatic experiments, we revealed that the age-related TAFs differences could result in the differences of epithelial-mesenchymal transition (EMT). Proved by both bioinformatic and cellular experiments, we confirmed that there were more samples could be related to mesenchymal subtype of GBM in equal and greater than 40 years old group than their under 40-year-old counterparts. And primary GBM cells from different aged patients also contained more spindle-like cells than those of under 40 years old, which indicated more mesenchymal cells in equal and greater than 40 years old samples. These results revealed a distinguishable link between age and TAFs, which may result in differences of incidence and prognosis in GBM patients. The specific mechanism behind this link may lead to further investigation for future targeting therapy.

## Methods and materials

### Data sources

#### Clinical data from the Surveillance, Epidemiology, and End Results (SEER) database (1975–2016)

Adult glioblastoma (GBM) data were downloaded from SEER database (Data Incidence-SEER 18 Regs Custom Data, with additional treatment fields, Nov 2018 sub 1975–2016 varying), using the SEER*Stat software, version 8.3.6. According to file description document (SEER RESEARCH DATA RECORD DESCRIPTION CASES DIAGNOSED IN 1975–2016), the filtering criteria were set as following: (1) CS Schema v0204 + code was “012 brain”; (2) Histology recode—Brain groupings code was “03 Glioblastoma”; (3) Age at diagnosis was not less than 18 years old. Finally, 61,997 GBM cases were screened out for further epidemiological analysis. When analyzing the primary site of the tumors, we deleted the data with unclear site records, “Primary Site—labeled” coded as: “C71.0-Cerebrum” and “C71.9-Brain, NOS”. 54834 GBM data were filtered at the end. Furthermore, in order to evaluate the prognosis of GBM, we excluded the cases with more than one tumor, and selected cases with diagnosis of GBM only. Moreover, cases with non-tumor related death causes were also excluded. Patients who were treated with biopsy or autopsy (coded as 00 in the datasets: “None; no surgery of primary site; autopsy ONLY”) without radiotherapy and chemotherapy were named as natural progression group; and those who underwent surgical resection (the resection scope were total resection coded as 21: “Subtotal resection of tumor, lesion or mass in brain” and subtotal resection coded as 30: “Radical, total, gross resection of tumor, lesion or mass in brain” in SEER dataset) were named as the resection group. In general, total number of 4627 and 9116 GBM cases were screened into the natural progression group and resection group, respectively.

#### RNA expression and clinical data from TCGA and CGGA

TCGA glioblastoma multiforme (GBM) gene expression data by AffyU133a array platform and clinical data were downloaded from UCSC Xena website (https://tcga.xenahubs.net). Data were standardized by “affy RMA” method, then were transformed into log_2_- for further analysis. “somatic.maf.varscan” file of GBM was downloaded from TCGA (https://portal.gdc.cancer.gov/) and was used to calculate Tumor Mutation Burden (TMB) score. Data from Chinese Glioma Genome Atlas (CGGA) website (https://www.cgga.org.cn/) were used as test and verification of the findings in mining TCGA [21–24]. RNA-seq libraries were sequenced by the Illumina HiSeq 2000/2500/4000 Sequencing System, then FPKM (fragments per kilobase transcriptome per million fragments) method was used to quantify in CGGA part B dataset. Gene expression data from CGGA part C dataset were performed on all samples using the Agilent Whole Human Genome Array and normalized using GeneSpring GX 11.0 software. All patients included in this study were not less than 18 years old.

### Survival and COX regression analysis

Kaplan–Meier analysis with log-rank test was used for the survival analysis. The “survminer”, “survival” R packages loaded in R software were used for survival analysis, COX regression analysis, as well as the visualization of these analysis. The “rms” package in R was used to build a nomogram model, and the data of model was used to verify the prediction effect of the model with bootstrap method (B = 1000). p < 0.05 was considered as significance.

### The evaluation of tumor microenvironment related cells

In order to evaluate the ratio of immune-stromal component in tumor microenvironment (TME) of each case, “ImmuneScore (representing the infiltration of immune cells in tumor tissue), StromalScore (captureing the presence of stroma in tumor tissue), and ESTIMATEScore (inferring tumor purity, negatively correlated with tumor purity)” were calculated by the “estimate” R package. The “MCPcounter [25, 26]” package in R was used to calculated the scores of microenvironment cells.

### Gene set enrichment analysis (GSEA) and the quantification of epithelial mesenchymal transition (EMT)

TCGA GBM cases were divided into two groups according to age (18–39 years and equal and greater than 40 years old) for GSEA analysis with the software GSEA 4.0.3 [27, 28]. Hallmark gene sets collection as the target sets were downloaded from the Molecular Signatures Database (MSigDB) to show the statistically comparison between the two groups. Gene sets with nominal p value < 5% and FDR < 25% in GSEA results were considered as the standard of significantly enriched pathways. Based on the “HALLMARK_EPITHELIAL_MESENCHYMAL_TRANSITION” gene set from MSigDB database, we calculated the EMT score with the methods of ssGSEA (single-sample GSEA) and arithmetic mean [29], then the results were standardized (with the method of (expression- minimum)/(maximum- minimum) and log_2_ transformed, respectively). The ssGSEA was carried out by “GSVA”, “GSEABase” and “limma” packages in R. The “plotROC” R package used to produce ROC curve (receiver operator characteristic curve, ROC) evaluating the diagnostic value of EMT score for mesenchymal type of GBM.

### Other bioinformatic analysis

Differentially expressed genes (DEGs) between the two groups (< 40 years group vs ≥ 40 years group) were selected by the “limma” R package with the absolute value of log_2_( fold change) > 1 and adjust p-value < 0.05. Intersected with GSEA analysis results, 29 DEGs were screened out and used for further analysis. Lasso (Least absolute shrinkage and selection operator) was used to shrink variable set by the "glmnet" package (family = "cox") in R. The “randomForest” R package was used to calculate the MDG (Mean Decrease in the Gini index), which used for evaluating the contribution of the 29 DEGs to the classification (< 40 years group vs ≥ 40 years group). The “pheatmap” R package was used for cluster analysis and heatmap with the DEGs. The correlation between two variables was calculated by “ggstatsplot” package in R with the methods of “spearman”. The Wilcoxon test was used as statistical method to compare the difference between two samples. And p < 0.05 was considered significant. ROC curves, percentage charts, and histograms were produced by “survivalROC”, “ggstatsplot” and “ggplot2” packages in R. Line charts were produced by Excel software. The version of R software is 3.6.3

### Culture of primary glioblastoma cells

Briefly, jelly-like tumor tissue was obtained during surgery, and removed into a sterilized 50 mL centrifuge tube with ice-cold Dulbecco's Modified Eagle Medium (DMEM) medium (Life Technologies Corporation) in it. Then the tumor tissue was carefully transported from operating room to laboratory in a clean icebox. Discard the supernatant, place the tissue sample in a sterile dish, and cut it into 1mm^3^ pieces with sterilize scissors and tweezers. Then collect the cut sample into a 15 ml centrifuge tube, add PBS with 1% penicillin–streptomycin (Gibco), mix and shake up and down for three times in order to remove the remaining red blood cells as thoroughly as possible. After the upper layer of liquid is clear, carefully remove the supernatant, add about 3 ml 0.25% Trypsin–EDTA (Gibco) for every 2cm^3^ tissue, incubate at 37 ℃ for 10 min, and shake it every 2 min to make the tissue fully digested. After the digestion, the upper fluid would be turbid, let the tube stand for 2 min, then move the supernatant into an Eppendorf (EP) tube. Centrifuge the EP tub for 5 min with 900 g, and resuspended the pellets in a culture disk with DMEM with 10% fetal bovine serum (Gibco, Thermo Fisher Scientific Inc.). Incubate under a temperature of 37 °C and 5% CO_2_. Medium was changed every 2 days. Primary GBM cells were irregular spindle-like cell under microscope. All participants read and signed an informed consent document with the description of the testing procedures approved by the ethical committee of the Sanbo brain hospital capital medical university (SBNK-YJYS-2020-007-02), and conformed to standards for the use of human subjects.

### Western blot

Western blot assay was conducted with primary GBM cells separated from patients and cultured for two passages. Total amount of 50 mg protein in each group were separated on 10% SDS-PAGE, then transferred to a 0.22 mm PVDF membrane (Millipore). The membranes were blocked with 5% skimmed milk at room temperature for 2 h, and then incubated with specific primary antibodies at 4 °C overnight. The membranes were incubated with appropriate HRP-conjugated secondary antibodies diluted at 1:5000 (Boster) at 37 °C for 1 h. Protein bands on the membrane were visualized with ECL Kit (Millipore) using FluorChem FC system (Alpha Innotech Corporation).

### Transwell assay

According to the manufacturer’s protocol, cell migration assays were conducted using a transwell system that incorporated a polycarbonate filter membrane with a diameter of 6.5 mm and pore size of 8 μm (Corning, NY). Total number of 1 × 10^4^ cell suspension in serum-free culture media was added to the inserts, which was then placed in the well of a plate filled with culture media containing 10% FBS (used as a chemoattractant). After 24 h of incubation at 37 °C, the non-migrated cells were removed from the upper chamber by wiping with cotton-tipped swabs, and filters were fixed with 4% paraformaldehyde for 30 min. The filters were then stained with a 0.1% crystal violet solution for 30 min at room temperature. Three fields of adherent cells in each well were randomly photographed under inverted microscope.

## Results

### Incidence differences in different aged GBM patients

As showed in flow chart in Fig. 1, 61,997 GBM cases (ranging from the year of 1975 to 2016) from the Surveillance, Epidemiology, and End Results (SEER) database were selected to conduct an epidemiological research. The range of age at diagnosis was 18–101 years old (63.27 ± 13.69), with a median age of 64 years old. A significantly sharp increasing of GBM incidence was observed among patients between 35 to 40 years old, while the incidence of GBM patients aged from 18 to 35 years old only presented slight and gentle increasing trend (Fig. 2a). To systematically investigate the age-related data from SEER, gender and tumor site distribution characteristics among differently aged patients were further evaluated. As showed in Fig. 2b and Additional file 1: Table S1, the general ratio of male to female incidence was 1.36:1 (ranging from 1.47 to 1.75 among the patients under 50 years old, then the proportion of female increased among patients over 50 years old). Moreover, tumor site distributions among GBM patients of different ages also revealed specific characters. Frontal lobe accounted for the largest proportion of all cerebral lobes in the GBM primary site (15941cases, 29.07% of total), followed by the temporal lobe (14,562 cases), overlapping lesion of brain and parietal lobe (10,618 cases and 10,035 cases), occipital lobe and other parts (including brain stem, cerebellum and ventricle). The proportions of temporal lobe among patients under 40 years old were significantly lower than those among patients equal and greater than 40 years old (Fig. 2c, d, Table 1 and Additional file 1: Table S1). The detailed distribution of gender and primary site were provided as Table 1.

**Fig. 1:** Flow chart showed the detailed information of mining the epidemiology data from SEER database

**Fig. 2:** Epidemiology analysis in SEER database presented a clear correlation between age and incidence of GBM. **a** The incidence of GBM patients in SEER database showed a specific age-related distribution character. The grouped histogram showed the incidence from 18 to 101 years old in SEER database, with the interval of 5 years (18–20, 20–25, 25–30, 30–35, 35–40, 40–45, ……, −100 +). From age of 18–35, the incidence of GBM patients increased slightly with age from 18 to 35, while the trend dramatically increased at the age from 35 to 40 years old. **b** Ratio chart presented the incidence of male and female patients among different ages. Male patients accounted for a relatively larger proportion of the total number of incidence in all age groups from 18 to 80 years old, but the proportion gradually decreases with age, and after 80 years old, the ratio of men to women is close to 1:1, and even more women patients over 80 years old were involved than men. **c**, **d** Ratio chart and line chart showed the tumor-site distribution characters among patients with different ages

**Table 1:** Characteristics of age at diagnosis in the sex and the cerebral lobes

Variable	Number	Age at diagnosis			
		Range	Mean ± SD	Median	Quartile(Q1–Q3)
Sex					
Male	35,690 (57.57%)	18–101	62.36 ± 13.60	63	54–72
Female	26,307 (42.43%)	18–101	64.50 ± 13.72	66	56–75
Primary site—labeled					
Frontal lobe	15,941 (29.07%)	18–99	63.75 ± 13.56	65	55–74
Temporal lobe	14,562 (26.57%)	18–101	63.69 ± 13.70	65	55–74
Parietal lobe	10,035 (18.30%)	18–98	62.93 ± 13.87	64	54–73
Occipital lobe	2557 (4.66%)	18–98	63.57 ± 13.85	64	55–74
Ventricle, NOS	282 (0.51%)	18–96	63.15 ± 13.76	64	56–73
Cerebellum, NOS	442 (0.81%)	20–94	63.01 ± 13.50	64	54–72
Brain stem	397 (0.72%)	20–94	61.89 ± 14.17	63	54–72
Overlapping lesion of brain	10,618 (19.36%)	18–101	62.20 ± 13.66	64	54–72

### Prognostic differences among GBM patients of different ages

To further elucidate the age-related distribution of GBM patients in detail, we then analyzed the prognosis of these patients that treated with (total resection and subtotal resection) or without (autopsy without radiotherapy and chemotherapy, termed as the natural progression group) resection interventions in the SEER database and radiotherapy or chemotherapy. In order to evaluate the age-related outcome differences, the GBM patients were then divided into groups by 10 years intervals of age. We noticed that the outcome of GBM patients under 40 years old were significantly better than their equal and greater than 40 years old counterparts. No statistically differences were observed between patients of 18–29 years old and 30–39 years old. In order to further validated these phenomena, patients were divided into two groups by age, namely under and equal and greater than 40 years old. We revealed that in both the natural progression group and resection group, 40 years old was the cut-off value for glioblastoma. The median survival OS were 2 months in under 40 years old group (95% CI 0.130–3.870) and 1 month in equal and greater than 40 years old group (95% CI 0.945–1.055) in the natural progression group; while in the resection group, the median survival OS were 27 months in under 40 years old group (95% CI 23.894–30.106) and 12 months in equal and greater than 40 years old group (95% CI 11.664–12.336), respectively (Fig. 3a, b). ROC curve of 3-, 6-, 12-month in natural progression group, as well as 12-, 24- and 36 months in resection group were produced. AUC values in the natural progression group were 0.632, 0.702 and 0.770 respectively. And in the resection group, the AUC values were 0.692,0.682 and 0.703 respectively (Fig. 3c). Thus, age was confirmed as an important risk factor on the outcome of GBM. To verify the impact of other risk factors on the prognosis of GBM, COX regression analysis was performed with the factors of sex, age at diagnosis, tumor location, tumor size, resection range, radiotherapy and chemotherapy or not in the resection group. As showed in the nomogram and COX regression result, the C-index value for the predicted OS was 0.684 (Additional file 2: Figure S1A, B).

**Fig. 3:** Age is an independent risk factor for the prognosis of GBM. **a** Patients treated with surgical intervention were divided into 7 groups based on age (18–29, 30–39, 40–49, 50–59, 60–69, 70–79, 80–95 years old, respectively). Kaplan–Meier (KM) curved (left side) showed better prognosis among patients aged with 18–39, compared to that of patients aged from 40–95 years old. Log-rank test was used as statistical method. *P* < 0.0001. KM curve on the right side showed the patients under 40 years old had significantly better prognosis than those equal and greater than 40 years old. Log-rank test was used as statistical method. *P* < 0.0001. **b** Patients in natural progress group (treated with non-resection intervention) were also divided into 7 groups based on age. KM curved (left side) showed better prognosis among patients aged with 18–39, compared to that of patients aged from 40–95 years old. Log-rank test was used as statistical method. *P* < 0.0001. KM curve on the right side showed the patients under 40 years old had significantly better prognosis than those equal and greater than 40 years old. Log-rank test was used as statistical method. *P* < 0.0001. **c** ROC curves showed age as a prognostic predictor and indicator of GBM patients both in the natural progression group. ROC curves of 3, 6, and 12 months were produced in natural progress, the AUC value of these ROC curves were 0.632, 0.702 and 0.770, respectively. ROC curves of 12, 24 and 36 months were produced in resection group, the AUC value of these ROC curves were 0.692, 0.682, and 0.703, respectively

### Age-related difference of Tumor Mutation Burden (TMB) and the components in Tumor microenvironment (TME)

Tumor mutation burden (TMB) could reflect the type and number of surface antigens of tumor cells, and thus can be used as an important indicator of tumor immunogenicity. It had been reported that TMB could be alternated with age. In order to confirm whether age could affect tumor immunity by regulating TMB, further experiments were then conducted. The mutation data of GBM patients were downloaded from the TCGA database for calculating TMB. It was revealed by correlation curve in Fig. 4a that TMB was positively correlated with age (p < 0.001, r = 0.31). Furthermore, as it was showed in Fig. 4b, the median values of TMB in patients under and equal and greater than 40 years old were 0.81 and 1.19, respectively (log_e_ (Wilcoxon) = 8.99, p < 0.001). Stromal cells and immune cells were the two of the most important components in TME. The level of these immune components was then evaluated by different bioinformatic methods. Patients equal and greater than 40 years old had higher stromal scores and ESTIMATE scores than the patients under 40 years old confirmed by data from different datasets. In the TCGA dataset, the media stromal scores were -106.51 in the patients under 40 years old against 135.84 in the patients equal and greater than 40 years old (log_e_ (Wilcoxon) = 9.62, p = 0.035) and the ESTIMATE scores were 694.09 and 1121.96 (log_e_ (Wilcoxon) = 9.61, p = 0.048) separately in patients under and equal and greater than 40 years old. Data in the CCGA datasets also showed consistent results with TCGA. No significant difference of immune scores were observed between the two groups, in TCGA and CGGA mRNA array GBM dataset and CCGA mRNA seq primary GBM dataset. But in CGGA mRNA seq recurrent GBM dataset, the immune scores were higher in the patients equal and greater than 40 years old (-98.24 vs 440.18, log_e_ (Wilcoxon) = 7.41, p = 0.002) (Fig. 4c).

**Fig. 4:** Factors related to tumor microenvironment (TME) differed significantly between patients under and equal and greater than 40 years old. **a** Correlation curve revealed a positive correlation between age and the level of TMB. Spearman test was used as statistical method. r = 0.31, *P* < 0.001; **b** Violin plot showed significantly higher level of TMB in patients equal and greater than 40 years old than those in patients under 40 years old. Wilcxon rank sum test was used as statistical method. log_e_ (Wilcxon) = 8.99, *P* < 0.001; **c** Violin plot showed the different level of immune score, stromal score and ESTIMATE score between groups of patients under and equal and greater than 40 years old by analyzing data from microarray data in TCGA (TCGA- microarray), microarray data in CGGA (CGGA- microarray), primary GBM RNAseq data in CGGA (CGGA-RNAseq-pGBM), recurrent GBM RNAseq data in CGGA (CGGA-RNAseq-rGBM). Wilcxon rank sum test was used as statistical method. log_e_ (Wilcxon) and P were provided on the right corner of each images

### Tumor associated fibroblasts (TAFs) was closely related to the incidence and prognosis among GBM patients of different ages.

To further clarify the underlying mechanism contributing to the difference in prognosis of different ages, we conducted further experiments. Total number of 29 differentially expressed genes (DEGs) were screened out by GSEA and differential gene expression analysis between the groups of patients over and under 40 years old (Additional file 3: Table S2). Correlation between TME constituents and DEGs were then evaluated. As showed in Fig. 5a, b, stromal cells, composed of endothelial cells and tumor associated fibroblasts (TAFs), were significantly correlated with some of the DEGs (p < 0.05), while no significant correlation between the immune cells (T cells, CD8 T cells, cytotoxic lymphocytes, NK cells, B lineage, monocytic lineage, myeloid dendritic cells, and neutrophils) with DEGs (p > 0.05). Moreover, further analysis showed that the level of TAFs showed obvious difference between the two groups, which was 6.39 in the patients under 40 years old, and 6.86 in the patients equal and greater than 40 years old (log_e_ (Wilcoxon) = 9.71, p = 0.001), however, there was no significant difference in the level expression of endothelial cells (Fig. 5c). The level of TAFs was also negatively correlated with the prognosis in patients of different groups. We found that lower level of TAFs had longer median OS time of 454 days, than that in higher level (404 days) (cut off value of TAFs = 6.32; p = 0.017) (Additional file 4: Figure S2 and Fig. 5d). Moreover, some of DEGs had most obvious correlation with the level of TAFs. For example, as showed in Fig. 5e, the expression of TAGLN was the most correlated genes with the level of TAFs (correlation coefficient = 0.72, p < 0.001).

**Fig. 5:** Tumor associated fibroblasts (TAFs) is a potential mechanism behind age-related prognosis difference of GBM patients. **a** Correlation plot showed the relation between main constituents in tumor microenvironment and DEGs. 6 DEGs were significantly correlated with stromal cells. While no DEGs were significantly correlated to immune cells. **b**, **c** Heat map showed the correlation among components stromal cells (endothelial cells and fibroblasts), age and DEGs. It showed in box plots that fibroblasts were more enriched component among patients equal and greater than 40 years old than those in patients under 40 years old. **d** Kaplan–Meier curve showed that patients with higher level of fibroblasts (showed in red) had significantly worse outcome than those with lower level of fibroblasts (showed in blue). Log-rank test was used as statistical method. *P* = 0.017. **e** Correlation plot showed the DEGs mostly correlated with fibroblasts. Among these genes, TAGLN, POSTN, TIMP1, SERPINE1 and NNMT was the top five genes mostly correlated with the level of fibroblast

### Epithelial mesenchymal transition (EMT) was the most enriched hallmark among different aged GBM patients

GSEA analysis showed that the gene expressions of the two groups (under 40 years old vs equal and greater than 40 years old) were significantly enriched in the EMT pathway (the NES was -1.60 (NOM p value = 0.027, FDR q value = 0.053)) and there were the largest number of DEGs in the EMT pathway (Fig. 6a–d). 10 genes related to prognosis were selected by LASSO-COX analysis from the 29 DEGs (Fig. 6e, f). 7 genes with MDG (Mean Decrease in the Gini index) values greater than 4 were considered to mostly contribute to the classification of the two groups (under 40 years old group and equal and greater than 40 years old) (Table 2), and they were included in the prognosis-related genes screened by LASSO-COX analysis. These genes were then divided into high and low expression groups by the cut off points (Additional file 5: Figure S3A–G). The Kaplan–Meier survival analysis suggested that the median survival time of the low expression groups were significantly longer than those of the high expression groups (p < 0.001) (Table 2). It was revealed that the expression of these genes in the patients under 40 years old were significantly lower than those in the patients equal and greater than 40 years old (Fig. 6g). Inspired by multiple researches, the EMT score was conducted by the method of ssGSEA [29] (referred as EMTs) and arithmetic mean with the EMT-related gene expressions based on the EMT gene set in the HALLMARK pathway, (performed in log2 scale, EMTs-mean). ROC curves revealed that this EMT scores could function as a feasible tool to quantify the level of EMT(Correlated pAUC was 69.5% (85–100% SP) and 75.8% (85–100% SE), respectively), with a strongly positive relation between two methods (R = 0.84, *P* = 2.2e–16) (Fig. 7a, b). The cut off points of EMTs expression level was 0.5 (Additional file 6: Figure S4). Low score of EMTs score had longer median OS (503 days vs 406 days, p < 0.001) (Fig. 7c). Moreover, it was also revealed that the EMTs was strongly correlated to TAFs (r = 0.81, p<0.001) (Fig. 7d) in TCGA dataset.

**Fig. 6:** Differentially expressed genes (DEGs) showed epithelial mesenchymal transition (EMT) as potential mechanism for prognosis differences between two age group. **a** Hallmark of enriched pathways related to cancer development were evaluated. Epithelial-mesenchymal transition (EMT) is the most enriched pathway among all. **b** Gene-set enrichment analysis (GSEA) analysis also showed significant enrichment among patients under and equal and greater than 40 years old. **c** Volcano plot showed total number of 29 DEGs overlapped between GSEA and DEGs. 14 genes related to EMT were showed in darker color. **d** LASSO regression further screen prognosis-related genes from the DEGs. Tuning parameter (lambda) screening in the LASSO regression model. The partial likelihood deviance was generated versus log(lambda), and the lowest partial likelihood deviance corresponded to the optimal number of genes. The dotted vertical lines corresponded to the optimal lambda value according to the 1 standard error criteria and the minimum criteria. When 10 genes remained, the partial likelihood deviance was the lowest. **e** The LASSO coefficient profiles of the 29 genes. A vertical line was drawn at the value chosen by tenfold cross-validation, which indicated that 10 non-zero coefficients were identified by the optimal lambda value. **f** The expression level of the 7 genes screened out by Lasso regression analysis was significantly higher in patients equal and greater than 40 years old (≥ 40 y, red color) than those in patients under 40 years old (< 40 y, blue color). Wilcxon rank sum test was used as statistical method. **, P < 0.01; **g** Differentially expressed genes among patients over (≥ 40 y, showed in red) and under 40 years old (< 40 y, showed in blue)

**Table 2:** Random forest graph screening of genes with MDG > 4 (strong correlation with age factors)

Gene	Median OS	95% CI		MDG	p-value
EFEMP2				6.93	p < 0.001
high	394	363.17	424.84		
low	630	473.82	786.18		
PDGFA				5.75	p < 0.001
high	394	363.43	424.57		
low	728	488.00	968.00		
TIMP1				5.58	p < 0.001
high	394	363.02	424.98		
low	737	273.71	1200.29		
STEAP3				5.02	p < 0.001
high	399	365.74	432.26		
low	603	478.25	727.76		
LGALS3				4.71	p < 0.001
high	394	359.63	428.38		
low	772	364.64	1179.36		
CBR1				4.70	p < 0.001
high	404	372.00	436.00		
low	630	410.11	849.89		
EMP3				4.03	p < 0.001
high	399	368.89	429.12		
low	918	504.51	1331.49

**Fig. 7:** The level of fibroblasts were positively correlated with EMT. **a**–**c** The evaluation of the accuracy of EMT scores. ROC curve showed the estimation value of EMT score on the diagnosis of mesenchymal and non-mesenchymal subtypes. AUC = 0.862; The correlation between different method calculating the level of EMT. Kaplan–Meier curve showed patients with higher EMT score (showed in green) had worse outcome than those with lower EMT score (showed in yellow). Log-rank test was used as statistical method. *P* < 0.0001. **e** Data from different databases all showed the consistent positive correlation between fibroblast and EMT scores. Spearman test was used as statistical method. r = 0.81, 0.88, 0.61 and 0.78 in TCGA, CGGA array, CGGA RNAseq and CGGA RNAseq (recurrent GBM, rGBM), respectively

### Differences in subtype distribution and cellular pathology between patients under and equal and greater than 40 years old

GBM could be divided into at least three subgroups, namely proneural (PN), classical (CL) and mesenchymal (MES) subtypes. Among them, MES had the worst outcomes. The transition from the subtype of PN into MES was considered as proneural-mesenchymal transition process, namely EMT process in GBM, which was considered as the aggressiveness and progressiveness of GBM. In order to confirmed whether the EMT differences among patients under and equal and greater than 40 years old could result in the proportion of different subtypes and then result in different outcomes, further data mining was then performed. As showed in Fig. 8a, a distinct distribution of subtypes appeared among patients of different ages. Patients of 18–39 years old had the largest proportion of neural and proneural subtype, while the smallest proportion of MES subgroup. On the contrary, patients equal and greater than 40 years old, MES and CL subtypes gained a significantly increasing proportion, while the proportion of PN and neural subtypes decreased dramatically compared to patients under 40 years old. Considering the prognosis of subgroups, the subtypes were then divided into mesenchymal and non-mesenchymal group. It showed that the proportion of mesenchymal accounted for 12% among patients under 40 years old, while in the patients equal and greater than 40 years old, the proportion of mesenchymal accounted for 33% (chi-square = 9.64, p = 0.002). Grouped by the interval of every ten years old, the mesenchymal GBM in each age group accounted for higher ratios, when the age was more than 40 years old. And the proportion of mesenchymal GBM increased significantly after the age of 40 (Fig. 8b).To verify whether the difference of TAFs was the potential mechanism of the subtype distribution differences, the level of TAFs of mesenchymal and non-mesenchymal was then compared and showed that higher level of TAFs in mesenchymal group compared to non-mesenchymal group (log_e_ (Wilcoxon) = 10.69, p < 0.001) (Fig. 8c). These results correspond to the previous conclusions, that was, age differences could cause differences in TAFs, which affects the distribution of GBM subtypes, and in turn leads to differences in prognosis. It was reported that TAFs functioned as frame-like constituents in GBM both in vivo and in vitro, and contributed to the EMT process of many types of tumors. Thus, primary glioblastoma cells from clinical patients were used to conduct cellular experiments. It was showed in Fig. 8d, e, Transwell assay revealed that primary glioblastoma cells from patients under 40 years old had significantly greater migration capacity compared to those from patients equal and greater than 40 years old (p = 0.0019). Western blotting assay showed higher expression of mesenchymal markers such as Vimentin and CD44, but lower expression of proneural (epithelial) marker E-cadherin in equal and greater than 40 years old group (Fig. 8f, g).

**Fig. 8:** Subtype distribution differences showed that higher mesenchymal subtype in patients equal and greater than 40 years old. **a** Composition charts showed a specific subtype distribution character of mesenchymal and other subtypes among different aged patients. **b** Patients equal and greater than 40 years old had higher level of mesenchymal subtype than patients equal and greater than 40 years old. Chi-square test was used as statistical method. *P* = 0.002; **c** Violin plot showed mesenchymal subtype had higher level of fibroblasts than those of other subtypes. **d**, **e** Transwell showed greater migration capacity in patients equal and greater than 40 (≥ 40) years old than those of patients under 40 (< 40) years old. **f**, **g** Western blotting assay showed higher expression of mesenchymal markers Vimentin and CD44 and lower expression of epithelial marker E-cadherin in group of equal and greater than 40 (≥ 40) years old than those of patients under 40 (< 40) years old

## Discussion

Aging is believed to be one of the most influential risk factors during the development process of many types of cancers [30–32]. It seems quite reasonable that the incidence and malignance of tumors should be positively correlated with aging. However, researches have proved evidences that this correlation is not that simple as a linear relation [33]. It had been revealed by numerous epidemiological studies that the rate of age-related increase in cancer incidence varies with different cancer types [13, 34]. In GBM, even if the previous finding proved the age range from 40 to 60 is the most prevalent age of diagnosis among all patients [1, 35], there still lack of epidemiological studies that could systematically analyze the aging level and incidence trend among GBM patients. With the newly developed database of SEER [36], now we could conduct a large-scale epidemiological study over longer time span, in order to screen out the exact correlation between age and GBM. We discovered that in the age group of 18 to 35 years old, the incidence of GBM has only slightly increased, with a gentle upward trend. However, in the age group from 35 to 40 years old, the incidence of GBM has dramatically increased with a sharp trend. There were only slight but not significant age-related differences of incidence between genders, nor was there any significant differences changed with the primary site of tumors. Moreover, prognosis of GBM also showed its unique distribution characteristics among different ages. By conducting further investigations, we noticed that the age of 40 was clearly an obvious prognostic “watershed age” for patients with or without surgical intervention, which indicated that the difference in the prognosis of GBM patients over and under the age of 40 is affected by the tumor itself rather than the treatments they’ve taken. These findings not only validated and extended the results of past epidemiological studies, but also further highlighted this specific age, namely 40-year-old, being a potential factors that need to be further investigated, and also encouraged us to further elucidate whether age heterogeneity could indicate any detailed mechanisms which could lead to any significant influences on the occurrence and development of GBM.

Understanding the links between cancer and aging is more important than ever. However, the interplay of aging-associated changes that could impact on cancer initiation and progression is complex [13, 18, 31]. There are many possibilities which could contribute to the differences within incidence as well as prognosis among different aged GBM patients, such as DNA damage responses [37], endocrine changes [38], vascular and angiogenesis [39], immune responses [40], alternation differences in tumor microenvironments [18], etc. Moreover, Nicola Alessio et al. [41, 42]reported that aged cells could secrete inflammatory cytokines, proteases, and other factors (termed as senescence-associated secretory phenotype (SASP)), which could greatly contribute to the cancer growth arrest, senescence, or apoptosis processes of different tumors. Among these potential mechanisms, there must be one or more molecular, genetical or cellular changes that played a pivotal role in the process of aging-GBM-interplay. It is because that GBM are highly heterogeneous at the cellular, molecule and histological level [5, 7]. In our research, we firstly noticed that TMB gradually increased with age, and there was a significant difference in TMB between patients over and under 40 years old. This differences in TMB indicate that the number of gene mutations accumulated per mega-base increases in the GBM cells of patients equal and greater than 40 years old, so that new antigens can be produced and make it easier for them to be recognized by immune and other type of non-neoplastic cells within the microenvironment of GBM. The major non-neoplastic immune cell population in the GBM microenvironment includes cells of the innate immune system called TAMs, as well as the stromal cells such as TAFs. TAMs and TAFs are of great importance in several aspects of the tumor progression and chemotherapeutic processes of GBM [11]. It’s been reported that age-related immune alternations could cause landscape remodeling of the tumor microenvironment and initiate the invasiveness and aggressiveness of tumors, including GBM [43]. Therefore, heterogeneity of TAMs and TAFs may function as significantly distinguishable prognostic factors in GBM patients. We then decided to further exam the immune level between under and equal and greater than 40 years old by evaluating stromal score (that captures the presence of stroma in tumor tissue), immune score (that represents the infiltration of immune cells in tumor tissue) and ESTIMETE score (that infers tumor purity) using the data from TCGA and CGGA databases. We found that in patients equal and greater than 40 years old, stromal score was significantly higher than that in patients under 40 years old in these databases, which indicated that the content level of stromal cells was significantly different among patients of the two aged groups. Stromal cells associated to tumors were specifically referred to two type of cells, namely endothelial cells and fibroblasts. In order to detailly clarify the certain content of various cell components, we use microenvironment cell population counter (MCPcounter) method to estimate the content of cells more accurately. We discovered that TAFs was the only component that were significantly different between over and under 40 years old patients. Then we raised a question that what is the potential mechanisms by which TAFs could lead to the worse outcome in aged GBM patients?

Until now, there is still lack of researches focusing on the role of fibroblasts in the development of GBM. In other type of tumors, TAFs could regulate the biology of tumor cells and other stromal cells via cell–cell contact, releasing numerous regulatory factors and synthesizing and remodeling the extracellular matrix, and thus these cells affect cancer initiation and development [12, 20]. The recent characterization of TAFs based on specific cell surface markers not only deepens our insight into their phenotypic heterogeneity and functional diversity [10, 44]. There are multiple sources of TAFs based on different cell populations. Among them, the fourth and fifth sources of TAFs are epithelial or endothelial cells that are adjacent to cancer cells and undergo EMT and can be induced to express S100A4, thus becoming an initiator of progressiveness and invasiveness of tumors [45, 46]. EMT process is biologically similar with the aggressiveness of GBM. It has been reported by many related researches that TAFs can trigger the process of EMT by generating cytokines and chemokines and induce pathways such as TGFβ – SMAD signaling, etc. in many types of tumors [47–49]. In order to investigate if it is also the case in GBM, we conducted a correlation analysis of EMT and fibroblast using quantification of EMT score generated by comprehensive single sample gene set enrichment analysis (ssGSEA) method. We revealed that the content of fibroblast is positively correlated with EMT score in GBM with different datasets, which inferred that fibroblasts could influence the development of GBM by initiating the EMT process and then result in the differences of incidence and prognosis of GBM patients from over and under 40 years old.

Furthermore, in addition to high levels of inter-tumoral heterogeneity, GBMs also exhibit high levels of intratumoral heterogeneity. Characterization of the genome, epigenome, and transcriptome of GBMs has provided a higher-resolution picture of frequent alterations. Using the GSEA enrichment method, we screened out the DEGs and the pathways enriched among them. To our astonishment, these DEGs were all positively correlated with fibroblasts, and EMT was also the most enriched pathway of the DEGs between under and equal and greater than 40 years old patients. Therefore, valid evidences had proved that EMT process was the mechanism that could potentially link the worse outcome and age in GBM patients.

Unsupervised transcriptome analysis revealed four subtypes of GBM, termed as classical, mesenchymal, neural and proneural, which were tightly associated with specific genomic abnormalities [50]. Proneuronal tumors seem to be associated with a better outcome, whereas mesenchymal tumors are related to a poorer survival. Under certain circumstances, different subtypes could transform into each other. The transition from proneural into mesenchymal termed as proneural-mesenchymal transition (PMT), namely EMT in GBM [51–53]. We firstly discovered that significantly more MES but less PN subtype in equal and greater than 40 years old patients than those under 40 years old. Encouraged by these bioinformatic findings, we conducted experiments at cellular level. It had long been established that during EMT, epithelial cells acquire a spindle-shaped morphology and properties of mesenchymal cells, including increased motility and invasiveness and the expression of a broad spectrum of mesenchymal markers. We discovered that the primary GBM cell of patients equal and greater than 40 years old showed more spindle-like cells at a morphology level compared to those of under 40 years old patients. These findings could prove that there were possibly more MES subtype cells in equal and greater than 40 years old patients and then result in worse outcome. As for the mechanism of how TAFs could lead to EMT, there are many possibilities. Besides of the chemokines and cytokines, the more TAFs could increase the adhesion between brain fiber bundle and GBM tumor tissue and make it easier for tumor to develop along the fiber bundle, so that the tumor progresses to a more malignant direction. In order to elucidate these hypotheses, we would conduct related experiments in our future study.

In conclusion, in this study, we revealed an uneven outcome distribution among different aged GBM patients which could significantly divide into two groups, namely patients over and under 40 years old. Proved by a group of bioinformatic experiments, we find that the content of TAFs out of other type of immune and stromal cells, was significantly different between these two groups of patients, and this difference of TAFs was directly link to EMT process. Confirmed by cellular experiments, we found that more primary cells of MES subgroups and higher migration capacity of primary GBM cells in patients equal and greater than 40 years old. This study linked the epidemiology and tumor biology of GBM, and explains the prognostic differences of patients of different ages and the underlying mechanisms, and provides a new perspective and direction for future related research.

## Supplementary information

**Additional file 1: Table S1.** Proportions of sex and lobes in different age groups.

**Additional file 2: Figure S1.** A Multivariate analysis for GBM clinical factors in resection group. COX regression result showed that the factors of age at diagnosis, tumor location, tumor size, resection range, radiotherapy and chemotherapy or not were prognostic risk factors for GBM in the resection group and the factor of age at diagnosis contributed the most to the COX regression model, HR= 2.580 (95% CI 2.256–2.951). 1B Nomogram for predicting the 1-, 2-, and 3-year overall survival in resection group.

**Additional file 3: Table S2.** Differentially expressed genes.

**Additional file 4: Figure S2.** The best cutoff of TAFs for prognosis. The cutoff was 6.32.

**Additional file 5: Figure S3.** A–G The best cutoff of DEGs for prognosis. The cutoff of CBR1, EFEMP2, EMP3, LGALS3, PDGFA, TIMP1 and STEAP3 were 7.15,6.17,6.61,9.51,5.94,9.75 and 5.89, respectively.

**Additional file 6: Figure S4.** The best cutoff of EMTs for prognosis. The cutoff was 0.5.

## Data Availability

Adult glioblastoma (GBM) data were downloaded from SEER database (Data Incidence-SEER 18 Regs Custom Data, with additional treatment fields, Nov 2018 sub 1975–2016 varying), using the SEER*Stat software, version 8.3.6. TCGA array gene expression data and clinical data were downloaded from UCSC Xena website (https://tcga.xenahubs.net). The “somatic.maf.varscan” file of GBM was downloaded from TCGA (https://portal.gdc.cancer.gov/). CGGA RNA-seq and array gene expression data and clinical data were downloaded from CGGA (https://www.cgga.org.cn/) part B and part C datasets.
